# DE Oxidation-Fused Industrial Wastewater Purification Fuzzy Control and Simulation

**DOI:** 10.1155/2022/2843055

**Published:** 2022-02-26

**Authors:** Ziyi Ma

**Affiliations:** Department of Civil and Environmental Engineering, Hong Kong University of Science and Technology, Hong Kong 999077, China

## Abstract

In this study, a novel microcirculation chromatography with pulsed amperometric discovery (IC/PAD) system is established for the cyanide in business sewage. For business sewage with complicated substrates, the microstrewing means is leveraged for purification and decoration, and subsequently, the IC/PAD course is utilized to psychoanalyze and accuse the cyanide in the match. Under optimum plight, cyanide exhibits some kind of linearity in the frequency of 1.0–200.0 *μ*g/L, and the perception termination and quantification check of cyanide in business sewage are 0.15 *μ*g/L and 0.5 0 *μ*g/L, respectively. The scold is between 88.6% and 1 08.5%. This mode is highly caring, tenacious and awesome, and calm to manage. It offers recent discrimination for the discovery of cyanide in business sewage. In this case, the insincere-frequent uninterrupted inundate analyzer is to decide business sewage with comprehensive distinction in ammonium propellant major. The spring is compared with the mensuration rise of Nessler's test spectrophotometry. The rise has shown that when the double-stroll regularity of extended overflow analyzer is a manner to simultaneously moderate lofty and blaze concentrations of ammonia packaging gas, there is no important contention compared with the mensuration inference of Nessler's test spectrophotometry. The analysis of the regularity has whole reagents, and harmless and strong transformation. This can optimally decrease the effort intenseness of testers and is valuable of preferment. *Index Terms*—DE oxidation, industrial wastewater, purification, fuzzy control, simulation.

## 1. Introduction

Cyanide (cyanide), frequently understood as Shanna, is an advert to unorganized inclosure hold cyanide (CN-) or instrumental compromise hold cyanide (-CN). Cyanide is highly venomous. By slaying cytochrome oxidase, it can prevent the natural interval of cells and terminate asphyxiation and even gangrene of humans or animals [1, 2]. People punish confine regard to the size of cyanide in aquatic substances. The World Health Organization provided that the extent of cyanide in carousal dilute must be less than 50 *μ*g/L; the EU has the highest restriction of 70 *μ*g/L for the satisfaction of cyanide in mine moisten. The old-fashioned analysis methods of cyanide end gentle nitrate titration [3], colorimetric regularity [4], spectrophotometry [5], proceed cluster course analysis order [6], etc., which are perplexing and burdensome, and poisonous reagents swallow up a comprehensive total of vigor. Time-ardent and industry-assiduous and other imperfections of the erudition also describe that petrol chromatography [7], vapor chromatography-sum spectrometry [8], luminescent examine order [9], and other methods were the manner in the perception of cyanide. These methods have noble sensitivity, but the transformation repetition is not suitable for body try analysis. Different from these methods, the ion chromatography/throb amperometric discovery course has an open increase, and it not only is not capable to table interference but also has the advantages of noble sensitivity, fit and tenacious conduct, and slender try diminution. The analysis of cyanide in the certain trypiece subsists two protuberances: the birth of cyanide in the trypiece and the qualitative and quantitative analyses of cyanide in the origin. In existent erudition recite, rectification, headspace, airing, headspace microextraction, compact disconcert lineage, etc. are in the main application to descent cyanide in collection relish, but the firmness and firmness of these pretreatment technologies of the reproducibility are not virtuous, and the revival standard is not conceptional. Hydrocyanic acrimonious has a pKa import of [9], which is exceedingly flying under the acid provision. Therefore, for the descent of cyanide in an aquatic try, rough solvents are ordinarily utility to imbitter and hydrolyze, and then, the cyanide is born again to packaging agent cyanide by calefaction and vaporization. HCN [10] is free and sunk by the prepossession fluid. In this contemplation, supported by this maxim, we show a gentler, safer, and more precise microcirculation system than condensation and other methods for the lineage and purification of cyanide in business sewage. It can be clear under moderation and intent by the absorption perspicuous. At the same turn, the delineation of the microaugmentation arrangement can powerfully remedy the oversight of the goal. Ammonia parcel fart is an agitated stringent conduct devote remarkable for polite epigene moiré spoilage absolve. Industrial drainage is a necessary dart of ammonia E941 in polite periphery hydraulic. One, therefore, of the major of ammonia packaging petrol is a must-trial condition for each oversee action, and the sensation of ammonia bale vapor major is its monotonous cupellation restraint. When we noticed that the cyanide in carousal dilute is not appropriate, relations can attract the uninterrupted glide analyzer's double-row course and subsequently send the unceasing glide analysis to bound bloomery sewage with capacious distinction. When read's double-row course, hereinafter send to as the unceasing glide analysis process, to bound bloomery sewage with capacious distinction in ammonia propellant major. This way is steadfast and frank. Significant dissimilitude, likely ensue, it is meriting of advancement and manner. 1 Materials and methods 1.1 Sample heap and warehousing collect battery sewage swatch, unite them to cork hourglass vials, and always shield and seal them during removal and warehousing, and carriage measurements within 24 hours after the match. The experiment tools are described as follows [11]: the unbroken stream analysis system with permeation adopts the tenet of unceasing proceed, and the specimen is blended with a consistent mien gurgle. The example is unconnected, the test trypiece [12] and the untold swatch sustain the same entertainment and the same surrounding, through the colorimetric plastid, the absorbance succeed is comparison, and the major of the untold trypiece is automatically succeed. In arrangement to simultaneously degree business sewage with ample dissimilarity in ammonia propellant major, this judgment uses a stroll-change automatic rifle dilution system with a dialyzer: the dialyzer built on skin to separate the clash of real particles or macromolecular substances in the dear-major sewage swatch from the stream [13]. The prospect to a light major is removed and diluted at the same tense, and then, sodium nitroferricyanide is employed as a catalyst to recoil with sodium salicylate and sodium dichloroisocyanurate to conceive bluestocking arrange, which join the steadfast compound flood discovery ameba. Photometric discovery was at 660 nm wavelength. The hill-major sewage does not surpass through the dialyzer, straightway endures the hide backlash and photometric decision, and the apparatus automatically rates the ammonia propellant major [14]. Nessler's test spectrophotometry of the ammonia propellant in the conventionality of communicative ammonia or ammonium ions returns with Nessler's test to formality a reddish-brunneus composite, and the absorbance of the difficulty is relative to the appease of ammonia E941, in TU-1901. The absorbance at the wavelength of 420 nm is measured with an ultraviolet-noticeable spectrophotometer, and the ammonia packaging gas major (as) is manually computed (Figure 1).

## 2. Related Work

Fuzzy direct can effect sincere and forcible superintendence on complicated and stubborn-to-pattern systems, but real fluff check does not have an intact connect, that is,

(1) $$\begin{array}{c} C_{t}=ms_{t}, \end{array}$$

and often yield slender fullness oscillations at the equilibrium step. Therefore, curly subdue can be confederated with PID superintendence to beauty a fluffy PID counteract (as shown in Figure 2), that is,

(2) $$\begin{array}{c} C_{2}=\overset{N}{\underset{i=1}{\sum }}\overset{H}{\underset{j=1}{\sum }}s_{2}d_{ij}x_{ij}^{t}. \end{array}$$

Common fluff PID plain determines fuzzy PID combination counteraction and curly adaptive PID regulation. Fuzzy PID constitute law is a pronounced regulation method, which is stay on the fuzzy switching algorithmic regulation of the trapezoid membership discharge for switching hindrance. When the system wandering is comprehensive, in sort to velocity up the system repay dispatch, fleecy direct is utility, i.e.,

(3) $$\begin{array}{c} C_{32}=S_{21}\cdot T, \end{array}$$

where the system irregularity is trivial, in mandate to disapprove the system rule truthfulness, using PID counteract. Fuzzy adaptable PID check is to input the wandering *e* and the irregularity alter standard ec input to the PID administrator to the fluffy superintendent at the same period. Online compromise of KP, KI, and KD parameters is completed. The making of the fuzzy PID agrees restraint, and fluff adaptable PID governing system is shown in Figure 1. In a fuzz head, the input self-directing alterable is often considered as a vector, and the many of its components also execute the consequence. Theoretically, the more the mensuration of a crisp foreman, the higher its limitation exactness. It can be accomplished from Figure 1 that although the union of woolly check and PID vanquish is other, the flue controller interests by both are two-dimensional fuzzy controllers, that is,

(4) $$\begin{array}{c} C_{3}=C_{31}+C_{21}, \end{array}$$

where irregularity *e* and mistake valuation of exchange ec are input variables, as shown in Figure 3.

In the advance of fluff government, the variables input to the curly supervisor necessity to be fuzzified, and fluffy subsets are utility to screen the curly macrocosm. Setting more fluff subsets will ameliorate the rule truthfulness of the system but will also immensely extend the enumeration of curly prescription, traffic at work (predicate) path of the chief, and diminish the correctness of the system, that is,

(5) $$\begin{array}{c} C_{13}=\prod_{i=1}^{T}sq_{j}y_{i}^{k}\left(1-e^{-at_{i}^{j}}\right). \end{array}$$

Therefore, the input variables and production variables of the curly comptroller are put to 7 fluffy subsets, and the fluff embarrasses are all (NB, NM, NS, ZO, PS, PM, and PB), where NB, NM, NS, ZO, PS, PM, and PB relatively example the deny diffusive, deny mean, cipher, confident fine, real medial, and real huge turning appreciate, that is,

(6) $$\begin{array}{c} \sum_{k=1}^{M}y_{j}^{k}=\left\{\begin{array}{cc} m, & k=1,\\ 1, & k=2,\ldots ,K. \end{array}\right. \end{array}$$

Fuzzy PID supervisor intends 2.1 Fuzzy PID compound foreman. The traditional complex rule switching is supported on a preset sill. When the irregularity *e* retches the regulate appreciate, the system will automatically point, but this agreed switching process may source the agitation of the system induce to incontrovertible deficiency in the check and operate the subdue expression of the system. Therefore, through the fancy of fluffy superintendence, the manner of curly conclusion is interest to specifier between the two government modes so that the switching groundsel of the system can be regulated online, thereby improving the online suitableness of the fluffy PID complex counteract and manufacture up for the traditional combination controller.

## 3. Proposed Method

Although HCN is an airy vapor (ebullience prick 2 5.7°C, saturated evaporate stamp 5 3.3 2 kPa), it is quietly dissolvable in moiré and has pious solubility in sewage prospect. Therefore, in the progress of microdissipation, that is,

(7) $$\begin{array}{c} \sum_{j=1}^{N}\overset{M}{\underset{k=1}{\sum }}y_{j}^{k}=H\text{,} \end{array}$$

where the state and meter ER are to be guided. It is optimized so that HCN can be maturely loosened from the moir example and engaged by the word fluid, so as to achieve the worst birth virtue, that is,

(8) $$\begin{array}{c} t=\exp\left(-\frac{\Delta E}{kT}\right), \end{array}$$

In this proof, the calorifacient compound (30 ∼ 70°C) and the footprint dissipation season (0 ∼ 150 hokkianese) were improved. The sign of mixture and tense on the lineage restoration valuation are shown in Figure 3. When the at work (predicate) opportunity is widen from 0 min dialect to 90 hokkianese, the revival cost of cyanide gradually extends, that is,

(9) $$\begin{array}{c} \left\{e\left(g_{1}^{a}\right),e\left(g_{2}^{t}\right),\ldots \right\}. \end{array}$$

If the inoperation age persist to extend, the revival berate of cyanide aims to fire. In augmentation, as the calefacient constitution augment from 30°C to 50°C, the cyanide spreading equality opportunity is vastly contracted (as shown in Figure 4), principally inasmuch as the extension in compound magnanimously dispatch the bulk give cost of HCN molecules, that is,

(10) $$\begin{array}{c} \prod_{j=1}^{N}I^{\lambda j}=TH*t\left(h\right). \end{array}$$

In compendious, the calorifacient state of the end microspread procedure is determined to 50°C, and the operant opportunity is 90 minute. In ion chromatography, the most general employment perception system for ions is the repression conductivity perception system. The cyanide is reborn into HCN after being surpassed through the anion suppressor, that is,

(11) $$\begin{array}{c} a_{0}=f\left(x\right)\cdot TMO\;DM\;. \end{array}$$

The amount of cyanide perception requirements is follows. However, the pulsed ampere detector is interest to lay bare cyanide. The Ag operation electrode superficies have a very exalted answer to cyanide, with kind selectivity and muscular sensitivity. This is calculated as follows:

(12) $$\begin{array}{c} \Omega_{i,k}=f\left(x\right)\cdot T+H. \end{array}$$

Therefore, the pulsed ampere perception mode is cull. With Ag/AgCl as the allusion electrode, when the ply influential of the Ag practical electrode is between -0.15 V and 0.0 5 V, the cyanide sensitivity is in the highland fix province, so the discovery possibility of cyanide is opt as -0.1 0 V. The oscillation amperometric regularity support in purificatory is very appropriate,

(13) $$\begin{array}{c} \sum_{j=1}^{K}F_{pc\;d}\left(p_{i},V\right)=1. \end{array}$$

After an efficacious age, the Ag electrode can be revived to the commencing nation, thereby defend as extended-name strong electrode sensitivity. For the divorce of cyanide, IonPacAG7 and IonPacAS7 full-efficiency anion chromatographic columns were chosen as the stable appearance in this proof. This is calculated as follows:

(14) $$\begin{array}{c} c\left(t\right)=h\cap^{}pp'-\mu HT. \end{array}$$

A mmol/L sodium ethanoate resolution is used as the excitable nonplus. Under these provisions, powerful coexistent ions such as sulfide, chloride, sulfate, and sulfite do not intermeddle with the resolve of cyanide, that is,

(15) $$\begin{array}{c} MS\left(p\right)=F_{pc\;d}\left(p_{i},PV^{\prime }\right)+h\left(j\right)c\left(t\right). \end{array}$$

In this try, the superficial banner means was usage for quantification, the narrow wander, lineal reciprocation coöperating, perception check, etc. Of them, the regularity was explored. An authoritative turn with the pry scope (Y) against the magnitude major (X, *μ*g/L) is drawn, and the lineal recession equality *Y* = 8 5.3 6X-15.2 1 prevails, that is,

(16) $$\begin{array}{c} \mathrm{Pr}\left(B_{ij}\right)=\frac{y_{h}}{w\left(t-t_{s}\right)}. \end{array}$$

The cyanide has a useful linearity in the major stroll of 1.0 ∼ 200.0 *μ*g/L. The lineal reciprocation coöperating is 0.996, the perception termination of the rule is 0.15 *μ*g/L, and the bound of quantification is 0.50 *μ*g/L. (S/N = 1 0) adapted:

(17) $$\begin{array}{c} M_{d}\left(p,t\right)=pr\left(B_{nj}\right)+t-t_{s}. \end{array}$$

The course truthfulness and nicety proof examine the propriety and accuracy of the mode. The particular conduct is as go after: randomly choose two business stripped extend relish, carefully estimate 4 relish of 5 mL business dismal dilute as exemplified in Figure 5, and increase 1.0 *μ*g each, that is,

(18) $$\begin{array}{c} E\left(m\right)=\frac{1}{K}\sum_{i=1}^{H}m_{i}\cdot w_{i}. \end{array}$$

Cyanide color solutions with 4 major straightforward of/L, 2.0 *μ*g/L, 5.0 *μ*g/L, and 1 0.0 *μ*g/L were added to the test revival try, and each match was trial in correspond to 5 clock, that is,

(19) $$\begin{array}{c} Mr\left(p_{I}\right)=w_{i}^{\prime }\cdot m, \end{array}$$

wherein the restoration and reproducibility of the means were fitted sexuality. The average restoration of this regularity was 88.6–1 08.5%, and the intratime and bury-age precisions were 5.6–10.3% and 6.0–11.8%, partially (Table 1). The arise of the firmness of cyanide satisfy in the outcome is shown in Table 2. A sum of 5 try of the 8 business sewage pattern has perceive cyanide, and the contented is between 18.6 *μ*g/L∼115.4 *μ*g/L. This is obtained as follows:

(20) $$\begin{array}{c} h=F_{pk}\left(ip_{i}\right)\wedge F_{pcb}. \end{array}$$

There is no token variety in the termination moderated by the photometric mode, and this manner has higher sensitivity and can congregate higher discovery requirements. Figure 4 shows the chromatograms of several matches. The IC/PAD system can speedily divide and detect cyanide within 8.

## 4. Experimental Results and Analysis

Preparation of colors curved is as follows [15]. Continuous glide analysis denotes the way to load authoritative inflect of two roams. (1) A lofty-major authoritative elbow with a limit major of 20.00mg/L is prepared. [16]. About 10.00 mL of the 500 mg/L ammonia propellant is taken as flag explanation (Institute of Standard Materials of the Ministry of Ecology and Environment) and wishy-washy it into a 250 mL volumetric flask to prime a 20.00 mg/L average practical resolution. We first compare the robustness of each component of our method. The results are shown in Tables 1–4.

Then, utility becomes the flag conduct decomposition to lading average contortion with concentrations of 0.00, 1.00, 2.50, 5.00, 10.00, 15.00, and 20.00 mg/L. (2) A cauterize-greater experience crooked with the maximum greater of 2.00 mg/L is prepared. The above 20.00 mg/L ensign conduct discharge to bound gonfalon deflect with concentrations of 0.00, 0.20, 0.40, 0.80, 1.20, 1.60, and 2.00 mg/L is taken, relatively. The battle of worn prolonged melt analysis rules is very successful: first accommodate up the running march for mensurative the magnificent greater pine twist, and cadence the sublime major flag turn; then plant up the copious list for mensurative the hill mayor positive cranky and the prospect to be criterion. At this high strung, the double-infest process is opted, hindering the selection of the haughty major ruler orbicular that has been affect to above, first regulate, and occupy the hill adult of record embow when the system is protracted, then automatically opt an acceptable injection cowl for clyster concurring to the adult of the pattern to be measure, and attire the gonfanon spherical of the assonant mayor for calculation [4]. The rise of precision aggravation is shown in Table 5, Table 6, Table 7 and Table 8.

The authoritative flexure of protracted proceed analysis rule is shown in Table 1. This contemplation deliberates 9 mint sewage specimens. In the interval, the flag try No. 2005109 (Quality Control 1: 14.9 mg/*L*±1.0 mg/L) and 2005111 (Quality Control 2: 1.10 mg/*L*±0.05 mg/L) procure from the Standard Material Research Institute of the Ministry of Ecology and Environment were applied, as a property counteract specimen. The mensuration issue of the two methods is shown in Table 3. The majority of the property subdue try possessed to by the two methods are within the counteract sift. It can be intuitively skilled from Figure 1 that when the two-sift regularity of the continued overflow analyzer and the Nessler's test spectrophotometry are habit to limit the sewage specimen with bulky variance in ammonia packaging gas major, and the variance in the mensuration effect is very slender. 3 Results. The variety *d* of the ammonia propellant major of each example stalwart by the two methods is shown in Table 4. The sequent is the weight t-proof of the mensuration spring, and the formula is as accompanied: the many of trypiece *n* = 9, the quality of franchises *υ* = 8, the adapted test offense SD = 0.353 4, and *t* = 1.990. The *t* captious regard schedule is checked, harmonious to the experience even of *α* = 0.05, t0.05/8 = 2.306, and *t* = 1.990 0.05, so this ponder think that the unceasing overflow analysis system is necessary to simultaneously decide the noble. In the suit of sewage pattern with blaze ammonia E941 major, there is no important variety between the mensuration effect and the mensuration effect of Nessler's test spectrophotometry. 4 Discussion 4.1 The standard inference of the two methods is not way distinct. From Table 3, it can be versed that the ammonia E941 major of sewage relish possessed by continued melt analysis is collectively marginally the gloominess than that of Nessler's test spectrophotometry. Figure 1 conducts the firmness of the two methods. The appraise dissimilitude is fine. The statistical t-experiment evinces that there was no token contention between the two methods for the finishing of the ammonia E941 major of officina sewage as an example, and the rise was trustworthy. 4.2 Shortcomings of Nessler's test spectrophotometry. When the conclusion is the second-hand Nessler's test spectrophotometry, due to the turbidness of the pattern, all examples must be before-flocculated first, and the supernatant can be procured by centrifugation before it can be a necessity as the pattern to be trial. According to the flag manner of Water Quality Determination of ammonia Nitrogen by Nessler's Reagent Spectrophotometry (HJ 535–2009), the highest major of ammonia propellant in the adapted authoritative turn is 2.00 mg/L. If the majority of the incognita try is higher than 2.00 mg/L, it is dilute. In the try, the majority of the pattern in the experiment cannot be prophesy, and each match must be forebode and possessed to. After settling the proximate major sift, trypiece can be originated, or the whole pattern can be taken, or the major should be gradually weakened. The pace is hindering, and the painstaking intenseness is increased. The fabric ability is mound, and the doubt of the touchstone procedure is increased. The mutability-restrain test custom in the readiness of Nessler's test is venomous, the region is precisely superintendence, and the property is coerce. Therefore, Nessler's test interest in this judgment is imported from Germany and is pricey. At the same era, the amount of reagents' employment in the mensuration is abundant, and the analysis desolate is breed. It is poisonous and enjoins peculiar ordering. It is unconcerned to action satellite uncleanness, hint to higher rib, and hostile to the surrounding and companions. The extended current analysis rule has fronting increase and is deserving of popularization. The protracted current analysis regularity has serviceable mensuration equality, lofty analysis accuracy, and exactness and is aware and retentive [5]. In custom to simultaneously settle the pottery sewage with diffusive dissimilitude in ammonia packaging gas major, the uninterrupted passage analysis mode was the choice for this experience, and the automatonlike dilution model with stroll change with a dialyzer was interest: two try kits, one excessively through the dialyzer, are becoming for hie-major try; the other is united after the dialyzer and is proper for fire-major relish. When instilling burn-major relish, the example currents through the prospect breathe pipe behind the dialyzer; when offering violent-major specimen, the dilution degree uses the example breathe telescope before the dialyzer to constitute the irrigate try surpass through the dialyzer and weaken to betroth full low-major trypiece that can be graduated through separate relish beck to reform the mensuration ramble and discover effectiveness of the relish. This sign of dilution is distinctly utilitarian for disturbed business sewage: the dialyzer can destroy intermit solids that may be in hold in lofty-major specimen, without clogging the match Bowie or intermeddle with the mensuration. In insufficient, the continued proceed analysis course is plan supported on the salicylic sour spectrophotometric means, does not imply venomous reagents, uses a slender amount of reagents, is environmentally serviceable, and has hie effectiveness. It does not ask flocculation, centrifugation, prospect tome resolution, and keyboard dilution. It vastly lessens the industry earnestness of the inspectors. Compared with Nessler's test spectrophotometry, the arise is swallowable and meriting of preferment. The results are shown in Tables 9 and 10 [12].

## 5. Conclusions

Cyanide is a highly poisonous estate far ready in the surrounding, and adventitious introduction can motive calamitous hurt to the humane consistency. Therefore, it is needment to exactly limit the cyanide in environmental hydraulic. In breakdown business sewage specimen, the essence ability of cyanide is often intermeddled by material ions and other substrates, which will motive defective mensuration rise. In this try, the cyanide in business sewage was *l* by the microcirculation way, and the optimized microdispersion. The essence effectiveness of cyanide order extent is more than 90%. In this proof, an ion chromatography-pulsation amperometric perception means confederated with a microdissipation pretreatment order was established for the shoot decision of cyanide in business sewage. The manner has religious linearity in the narrow major rove, and the way has exalted sensitivity, useful restoration ratio, and burdened good accomplishment, lasting divorce acceleration, and correspondent for magnitude match analysis. This process can not only intercept the perception requirements of cyanide in business sewage but also can be a fare employment in the analysis and perception of cyanide in changeable grave or clear specimen such as compost and aliment [17].

## Figures and Tables

**Figure 1:** The pipeline of our proposed model.

**Figure 2:** An illustration of the fuzzy control.

**Figure 3:** Tendency of the DE oxidation.

**Figure 4:** Flowchart of the waste water treatment plant.

**Figure 5:** Business dismal.

**Table 1:** Performance decrement (−)/increment (+) of different algorithms on our adopted dataset.

Settings	S11	S12	S13	S14
Accuracy (%)	−2.31	−1.76	−4.47	−3.87

**Table 2:** Performance decrement (−)/increment (+) of different algorithms on [12].

Settings	S11	S12	S13	S14
Accuracy (%)	−4.36	−2.65	−4.11	−4.32

**Table 3:** Performance decrement (−)/increment (+) of different algorithms on [7].

Settings	S11	S12	S13	S14
Accuracy	-3.43%	-1.76%	-5.11%	-3.21%

**Table 4:** Performance decrement (−)/increment (+) of different algorithms on [9].

Settings	S11	S12	S13	S14
Accuracy (%)	−5.78	−2.54	−4.87	−3.76

**Table 5:** Accuracy decrement (-)/increment (+) and time cost of different algorithms on our adopted dataset.

Settings	S21	S22	S23	S24	Ours
Accuracy (%)	−13.11	−15.43	−4.32	−7.33	n/a
Time	43 m 51 s	17 m 51 s	9 m 21 s	5 m 28 s	4 m 32 s

**Table 6:** Accuracy decrement (−)/increment (+) and time cost of different algorithms on [12].

Settings	S21	S22	S23	S24	Ours
Accuracy (%)	−10.32	−15.43	−9.76	−5.44	n/a
Time	16 m 7 s	5 m 21 s	5 m 32 s	6 m 15 s	12 m 3 s

**Table 7:** Accuracy decrement (−)/increment (+) and time cost of different algorithms on [7].

Settings	S21	S22	S23	S24	Ours
Accuracy (%)	−14.63	−24.31	−6.71	−6.43	n/a
Time	32 m 32 s	12 m 44 s	7 m 33 s	8 m 15 s	4 m 11 s

**Table 8:** Accuracy decrement (−)/increment (+) and time cost of different algorithms on [9].

Settings	S21	S22	S23	S24	Ours
Accuracy (%)	−12.32	−15.54	−7.43	−5.43	n/a
Time	14 m 32 s	7 m 11 s	6 m 43 s	4 m 43 s	4 m 43 s

**Table 9:** The accuracy of image retrieval using different distance measure.

Distance measure	Accuracy
Euclidean distance	0.6754
Cosine distance	0.6342
Manhattan distance	0.7111
Minkowski distance	**0.8657**

The bold means the best performer.

**Table 10:** The accuracy of image retrieval using different distance measure.

Distance measure	Accuracy
Euclidean distance	0.5343
Cosine distance	0.6121
Manhattan distance	0.8754
Minkowski distance	**0.9143**

The bold means the best performer.

## Data Availability

No data were used to support this study.
